The article "The application of key feature extraction algorithm based on Gabor wavelet transformation in the diagnosis of lumbar intervertebral disc degenerative changes" was retracted in 2023. Reasons: unreliable results or conclusions; concerns about the peer review.

# The application of key feature extraction algorithm based on Gabor wavelet transformation in the diagnosis of lumbar intervertebral disc degenerative changes

**DOI:** 10.1371/journal.pone.0227894

**Published:** 2020-02-26

**Authors:** Tao Yang, Renzhi Li, Ning Liang, Jing Li, Yi Yang, Qian Huang, Yuedan Li, Wei Cao, Qian Wang, Hongxin Zhang

**Affiliations:** 1 Department of Pain Treatment, Tangdu Hospital, The Fourth Military Medical University, Xi’an, China; 2 The 31638 Troops of The Chinese People’s Liberation Army, Kunming, China; 3 Department of Radiology, The 75th Group Army Hospital, Dali, China; 4 Department of General Surgery, The 75th Group Army Hospital, Dali, China; 5 College and Hospital of Stomatology, Xi’an Jiaotong University, Xi’an, China; 6 Department of Obstetrics and Gynecology, The 75th Group Army Hospital, Dali, China; 7 Department of Pharmacy, General Hospital of Central Theater Command, Wuhan, China; 8 Department of Anorectal Surgery, The First Affiliated Hospital of Zhengzhou University, Zhengzhou, China; University College London, UNITED KINGDOM

## Abstract

**Objective:**

Based on the theoretical basis of Gabor wavelet transformation, the application effects of feature extraction algorithm in Magnetic Resonance Imaging (MRI) and the role of feature extraction algorithm in the diagnosis of lumbar vertebra degenerative diseases were explored.

**Method:**

The structure of lumbar vertebra and degenerative changes were respectively introduced to clarify the onset mechanism and pathological changes of lumbar vertebra degenerative changes. Most importantly, the theoretical basis of Gabor wavelet transformation and the extraction effect of feature information in lumbar vertebra MRI images were introduced. The differentiation effects of feature information extraction algorithm on annulus fibrosus and nucleus pulposus were analyzed. In this study, the data of lumbar spine MRI was randomly selected from the Wenzhou Lumbar Spine Research Database as research objects. A total of 130 discs were successfully fitted, and 109 images were graded by a doctor after observation, which was compared with the results of the artificial diagnosis. Through the comparison with the results of observation and diagnosis by professional doctors, the accuracy of feature extraction algorithm based on Gabor wavelet transformation in the diagnosis of lumbar vertebra degenerative changes was analyzed.

**Results:**

1. Compared with the results of the manual diagnosis, the accuracy of the classification method was 88.3%. In addition, the specificity (SPE), accuracy (ACC), and sensitivity (SEN) of the classification method were respectively 89.5%, 92.4%, and 87.6%. 2. The mutual information method and the KLT algorithm were utilized for vertebral body tracking. The maximum mutual information method was more effective in the case of fewer image sequences; however, with the increase of image frames, the accumulation of errors would make the tracking effects of images get worse. Based on the KLT algorithm, the enhanced vertebral boundary information was selected; the soft tissues showed in the obtained images were smooth, the boundary information of vertebral body was enhanced, and the results were more accurate.

**Conclusion:**

The feature extraction algorithm based on Gabor wavelet transformation could easily and quickly realize the localization of the lumbar intervertebral disc, and the accuracy of the results was ensured. In addition, from the aspect of vertebral body tracking, the tracking effects based on the KLT algorithm were better and faster than those based on the maximum mutual information method.

## 1. Introduction

With the development of society and the increased working pressure of people, spinal diseases have become a kind of common orthopedic disease that affects human health and normal life [1]. According to statistics, the incidence rate of spinal diseases in China over 50-year-olds has exceeded 95%. In addition, the onset of spinal diseases has shown a trend of youthfulness; 1 of 5 children would suffer from scoliosis [2]. Therefore, spine-related diseases have already jeopardized the health of all human beings and should be valued [3]. Of all the spinal diseases, lumbar vertebra degenerative disease is a common and frequently-occurring disease [4]. Its clinical manifestations include different degrees of lower back pains and nerve root compression symptoms [5]. It is currently believed that degenerative changes of the lumbar intervertebral disc are an irreversible pathological process in the aging process of humans. At present, the mechanism of lumbar vertebra degeneration changes has not been fully understood yet. It is certain that its occurrence is closely related to the reduction of lumbar stability, and certain physical and chemical factors would accelerate the process of degeneration [6].

Clinically, in the diagnosis of lumbar diseases, in addition to routine examinations, medical imaging is often required as a reference. With the rapid advancement of medical imaging technology, various medical imaging technologies such as computed tomography (CT), ultrasound (US), magnetic resonance imaging (MRI), and positron emission tomography (PET) have been greatly developed [7]. These medical imaging technologies play an important supporting role in the clinical diagnosis and treatments, which have been recognized worldwide [8]. However, at the same time, in the face of a large number of medical images, medical personnel need to manually observe and analyze the image data; not only the workload is significantly increased but also the diagnosis results are related to the personal experiences of doctors [9]. Which are often subjective and are likely to affect the diagnostic accuracy of diseases [10].

In terms of the information analysis and processing of frequencies and directions in the local region, the analysis of digital images by Gabor wavelet transformation has excellent performances and could localize the signals of the time domain [11]. Through the 2D or 3D processing of medical images, doctors are able to observe the digital images in multiple directions; by locating and segmenting the region of interest of the images, the qualitative and quantitative analysis of the lesion regions could be achieved, which could improve the accuracy of clinical diagnosis and reduce the workload of doctors at the same time. In addition, doctors could analyze the dynamic parameters of lumbar motions by counting the results of continuous image sequence processing and understand the features of lumbar motions, which has important reference value for the diagnosis and treatment of lumbar intervertebral disc diseases [12]. In this study, the related algorithms of key feature extraction in Gabor wavelet transformation were discussed, and the localizing effects of feature extraction on intervertebral disc in lumbar diseases were analyzed.

## 2. Literature review

In China, the application of Gabor wavelet-based MRI images in the diagnosis of intervertebral disc disease has been confirmed by scholars through experiments. [13] proposed an unsupervised and fully-automated intervertebral disc localization and degenerative changes classification algorithm based on Gabor features; in addition, the MRI data of 37 patients were used for tests; the accuracy of the localization method was 96.6%, which could evaluate the degenerative changes of levels 1–5. Based on the objective MRI measurement of the intervertebral disc. [14] proposed a Gabor wavelet-based intervertebral disc localization algorithm, which used the gray ratio of the two and the height information of the intervertebral disc to achieve the classification of intervertebral disc degenerative changes. [15] found that MRI T2 mapping imaging technology could not only quantitatively assess the degree of lumbar intervertebral disc degeneration but also reflect the differences in the degenerative degrees of intervertebral discs in different levels through the T2 values of the nucleus pulposus, providing imaging basis for disease diagnosis. Through the clinical research, [16] found that CT and MRI had certain advantages in the clinical diagnosis of lumbar disc herniation, and the combined application of CT and MRI could reduce the rate of missed diagnosis if necessary.

Globally, scholars have achieved fruitful results in researching the MRI diagnosis of degenerative disc diseases, especially the MRI quantitative detection. [17] found that the intervertebral disc degeneration and multifidus amyotrophy were positively correlated at the L3-L4 intervertebral disc level, and the strengthening program of lumber intervertebral extensor muscle helped prevent amyotrophy and lumbar degeneration. [18] found that T2 and T1rho quantitative magnetic resonance imaging could detect the early degenerative changes of the intervertebral disc, and T1rho was more effective in the differential diagnosis of early degenerative diseases. Through clinical trials, [19] found that the early lumbar intervertebral disc degradation could be quantitatively evaluated by using MRI chemical exchange saturation transfer technique.

At present, in the field of MRI imaging detection for the diagnosis of intervertebral disc diseases, scholars have done a lot of researches. However, in terms of MRI image analysis, further research is needed to improve the extraction and analysis of images. Therefore, it is hoped that by applying the key feature extraction algorithm based on the Gabor wavelet, a more detailed analysis of lumbar disc degenerative MRI images would be made to improve the diagnosis of the disease.

## 3. Degenerative changes of the lumbar intervertebral disc and theoretical basis of Gabor wavelet transformation

### 3.1 The structure of lumbar vertebra and the degenerative changes

According to [14, 16, 20, 21]. The lumbar vertebra is a part of the vertebral column, which is located in the middle of the back and is made up of vertebrae and intervertebral discs. The vertebral column of an adult consists of 23 intervertebral discs and 33 vertebrae. The vertebrae include 7 cervical vertebrae, 12 thoracic vertebrae, 5 lumbar vertebrae, 5 sacral vertebrae, and 4 caudal vertebrae.

The annulus fibrosus is composed of a multi-layered fibrous cartilage annulus, which protects and limits the movement of the nucleus pulposus. Studies have found that the degenerative changes of the lumbar intervertebral disc are associated with decreased lumbar stability. At first, the stability of the lumbar vertebrae was only considered to be related to the structure of the vertebrae and the intervertebral disc. As people further explored the surrounding tissues such as muscles and ligaments, it has been found that the lumbar vertebrae, para-vertebral muscles, ligaments, and nerves jointly maintained the stability of the lumbar vertebrae. If any of these structures has a lesion, the compensation by other structures would be caused. When the compensation reaches the limit, a decrease in the stability of the lumbar vertebrae would occur. The unstable structure of lumbar vertebra could adversely affect the lumbar vertebra and its ancillary structures; in addition, if the unstable structure continues to exist without interventions, the vicious cycle would eventually accelerate the progression of lumbar intervertebral disc degenerative changes. According to [1,22,23], the main manifestations of lumbar vertebra degeneration are changes in the structures of the intervertebral discs, facet joints, muscles, and ligaments, in which the degeneration of the intervertebral discs is the basis and key manifestation of lumbar degenerative diseases, and lumbar disc herniation (LDH) is the most common disease.

LDH is due to the degeneration of the lumbar intervertebral discs, the rupture of the annulus fibrosus, the herniation and water loss of nucleus pulposus, and the loss of elasticity, which would result in the stimulation or compression of the nerve root and cauda equina in the corresponding segment and cause symptoms such as lower back pains, lower extremity radiation pains, muscle spasm, and limited mobility. Most LDH patients would choose conservative treatments to relieve the symptoms of pain; however, about 10% to 18% of LDH patients are in severe conditions, and surgical treatment must be taken to relieve the nerve compression. In terms of the surgical treatment, by cutting the intervertebral spaces of the lesions, the bone window, the adjacent lamina, and the medial articular process are excavated to completely decompress the pressures and improve the symptoms; currently, it is the most common surgical treatment for LDH, and its long-term therapeutic effects are satisfactory.

### 3.2 The theoretical basis of Gabor wavelet transformation

In the 20th century, Gabor proposed a method of expressing a time function by using both time and frequency. The equations represented by this method were called Gabor transformation. Gabor transformation is one of the optimal methods for image representation in signal processing. Based on the consideration of signal reconstruction stability, Gabor transformation is divided into two cases, i.e. the critical sampling and oversampling. The smallest changes in the lumbar intervertebral discs are the boundaries and the angles; thus, the Gabor wavelet transformation could be used to identify and localize the intervertebral discs through the information extraction of texture and angle.

Wavelet transformation is a kind of time-frequency analysis. It takes the wave functions of a certain energy that are concentrated in the time domain as the mother wavelet; through the scaling and translating of the mother wavelet, a specific base is formed; thus, the signals are transformed into progression series for multi-scale refinement analysis, and information could be extracted from the series. If a basic function φ(t) is given, which satisfies the condition $\int {}_{-\infty }^{\infty }\varphi (\text{t})=0$ as a basic wavelet function, it is assumed that:

$$\varphi_{\text{a},\text{b}}=\frac{1}{\sqrt{\text{a}}}\varphi (\frac{\text{t}-\text{b}}{\text{a}})$$ (1)

In the equation, a represents the scale factor, b represents the translation factor, and x(t) is the signal of the given square-integrable; the wavelet transformation expresses the signal x(t) as the projection superposition on the wavelet sequences obtained after the scaling and translating of the basic wavelet function:

$$\text{W}{\text{T}}_{\text{x}}(\text{a},\text{b})=\frac{1}{\sqrt{\text{a}}}\int \text{x}(\text{t})\varphi_{\text{a},\text{b}}^{*}(\text{t})\text{dt}$$ (2)

The essence of the Fourier Transform (FT) is to characterize the signals on the orthogonal basis of the trigonometric function. The spectral analysis method of this signal reflects the spectral features of the signals in the overall time and could better reveal the features of the stationary signals. However, since Fourier analysis uses global transformation, it cannot reflect the features in the local regions. For the common non-stationary signals that need to understand the local features of time-frequency, the FT has no advantages in signal representation. Compared with FT, wavelet transformation has the ability to characterize the local features of signals in both time and frequency. Wavelet transformation could realize the analysis of local features of time-frequency by adjusting the basic scale and displacement. Through the utilization of different steps of different frequencies in different time domains, wavelet transformation could perform local analysis in both time and frequency domains; it could completely display any details of the signals, thereby achieving the purpose of multi-resolution analysis.

In order to extract the features of an image P(x, y), its Gabor wavelet transformation could be defined as:

$${\text{W}}_{\text{mn}}(\text{x},\text{y})=\int \text{P}(\text{x},\text{y}){\text{g}}_{\text{mn}}^{*}(\text{x}-{\text{x}}_{1},\text{y}-{\text{y}}_{1})\text{d}{\text{x}}_{1}\text{d}{\text{y}}_{1}$$ (3)

In the equation, “*” indicates the complex number of conjugates. If the local texture region has spatial consistency, the mean number and standard deviation of its transformation coefficient are respectively expressed as Eqs (4) and (5):

$$\mu_{\text{mn}}=\int \int \left|{\text{W}}_{\text{mn}}(\text{x},\text{y})\right|\text{dxdy}$$ (4)

$$\sigma_{\text{mn}}=\sqrt{\int \int {\left({\text{W}}_{\text{mn}}(\text{x},\text{y})-\mu_{\text{mn}}\right)}^{2}\text{dxdy}}$$ (5)

The 2D Gabor transformation has good time-frequency localization features; it could extract the local detail features of different scales and directions on the images and has the ability to distinguish signals in space and frequency; thus, it could be used to extract salient features that are more suitable for recognition. The impulse response of a Gabor filter can be defined as a sine wave multiplied by a Gaussian function. Due to the multiplicative convolution property, the Fourier transform of the impulse response of the Gabor filter is the convolution of the Fourier transform of its harmonic function and the Fourier transform of the Gaussian function. The filter consists of real and imaginary parts, which are orthogonal to each other. A set of Gabor function arrays with different frequencies and directions is very useful for image feature extraction.

### 3.3 The classification algorithm for MRI images of lumbar intervertebral disc degenerative changes based on Gabor wavelet transformation

At present, the clinical diagnosis of lumbar intervertebral disc degenerative changes mainly depends on the image data of CT and MRI. In terms of the definition of lesion locations and extents, MRI has a higher contrast resolution and certain advantages. In terms of the MRI images of the intervertebral discs, the nucleus pulposus and annulus fibrosus of the normal intervertebral discs are significantly different in the T2-weighted images, the nucleus pulposus would show high-brightness signals while the annulus fibrosus would show low-brightness signals; with the onset and development of intervertebral disc degeneration, the differences between the signals of annulus fibrosus and nucleus pulposus gradually decrease; with the aggravation of degenerative degrees, the signal intensity of the nucleus pulposus gradually weakens and tends to be consistent with the brightness of the annulus fibrosus. [24] proposed an 8-level classification system of intervertebral disc degenerative changes in order to resolve the divergence among doctors in the judgment of certain indicators during the classification of moderate to severe intervertebral disc degeneration, as shown in Table 1.

**Table 1:** The 8-level classification system of intervertebral disc degenerative changes.

Classification	The signal intensity of nucleus pulposus and inner annulus fibrosus	The difference of fiber signal between inside and outside of the posterior annulus	Disc height
1	Homogeneous high signal, comparable to CSF signal	Obvious	Normal
2	High signal (stronger than presacral fat less than cerebrospinal fluid) or fissures in high signal nucleus pulposus	Obvious	Normal
3	High signal (less than presacral fat) Obvious	Obvious	Normal
4	Medium-high signal (slightly stronger than outer annulus)	Not obvious	Normal
5	Low signal (equal to outer ring)	Not obvious	Normal
6	Low signal	Not obvious	Reduction of <30%
7	Low signal	Not obvious	Reduction of 30%~60%
8	Low signal	Not obvious	Reduction of >60%

## 4. Experimental methods

### 4.1 Research objects

This study randomly selected lumbar spine MRI data from the Wenzhou Lumbar Spine Research Database as the research objects. This study was approved by the ethics committee of the hospital. Each volunteer participating in the lumbar spine study knew the research content and signed the informed consent forms.

Inclusion criteria: (1) Patients aged between 40 and 65 years; (2) Patients with symptoms of lumbar instability, symptoms of lumbar buttock pain and neurological damage related to lumbar spine movement (flexion, extension, lateral flexion, rotation) or posture change, including sudden movement restriction, “unstable interlocking” of the waist, which could be relieved through rest or brace braking; (3) Patients with no lumbar spondylolisthesis, structural scoliosis, severe osteoporosis, old fractures, and history of lumbar spine surgeries.

### 4.2 The analysis of intervertebral disc and the processing of image information

In this study, a total of 130 discs were successfully fitted, and 109 images were graded by a doctor after observation, which was compared with the results of the artificial diagnosis. Since the shape of the intervertebral disc approximates an ellipse, a more compact boundary could be obtained by fitting the boundary points of the ellipse. First, the Gabor filter was used to extract reliable boundary information to the maximum extent. Based on the accurate localization results, the wavelet coefficient map of the corresponding region in the localization coordinates was analyzed. By plotting the median Gabor coefficient map and analyzing the wavelet coefficients of the region in different directions, the general direction of the intervertebral disc at that position could be determined, i.e. the direction in which the mean intensity was maximized.

By analyzing the local region of the intervertebral disc, it could be determined that the elliptical fitting results were combined with the Gabor coefficient distribution, which was reasonable and feasible to distinguish the nucleus pulposus from the annulus fibrosus. Thus, the parameters of the gray-scale features of the two regions could be separately calculated to classify the degeneration of the intervertebral discs. The ratio of the gray values of nucleus pulposus to the gray values of annulus fibrosus was used as a parameter for characterizing the gradation characteristic to satisfy the different gradation parameters when the image gradation range was different. Fig 1 showed the effects of the differentiation between the nucleus pulposus and the annulus fibrosus by this method. It could be seen that the segmentation results were basically consistent with the actual tissues.

**Fig 1:** The differentiation of annulus fibrosus and nucleus pulposus. (a) The annulus fibrosus, (b) The nucleus pulposus.

The evaluation criteria for classification results of lumbar degenerative changes: respectively, the specificity (SPE), the accuracy (ACC), and the sensitivity (SEN) were used as evaluation criteria, which could be expressed as:

SPE=TN/(TN+FP) (6)

SPN=TP/(TP+FN) (7)

ACC=(TP+TN)/(TP+TN+FN+FP) (8)

In the equations, TP indicated the number of true positives in the test results, TN indicated the number of true negatives, FP indicated the number of false positives, and FN indicated the number of false negatives, where TP and TN were the conditions of illness or non-illness respectively confirmed by the detection standard and the tests. In terms of the lumbar degenerative changes, the classification results of professional doctors were used as the primary diagnostic standards. If the specificity of the diagnostic test was high, the misdiagnosis rate was considered to be lower; if the sensitivity of the diagnostic test was high, the proportion of missed diagnosis was considered to be less.

### 4.3 Measuring method of lumbar vertebral body movement

Image registration was the basis of image target tracking. By mapping the two images to each other, the points corresponding to the spatial locations were linked. In addition, the feature-based registration extracted the image feature information, established the correlation between the image and the floating image, and had the advantages of wide processing ranges and fast processing speed; the gray-based registration was based on the internal information of the images, the calculation of the grayscale statistics was performed to obtain the registration transformation parameters, which had higher precision and reliability.

1. Mutual information method: The degree of interdependence between two random variables was described by mutual information, which was generally expressed by entropy. The mutual information method in image registration meant that when two images with consistent content were registered by geometric transformation, their mutual information amount was maximized. It was supposed that two random variables were set as X and Y, p(x) denoted the probability density function of X, p(y) denoted the probability density function of Y, and p(x, y) denoted the overall probability density function of X and Y; then, the mutual information of X was expressed as S(x), and the overall mutual information of X and Y was expressed as S(x, y):
  $$\text{S}(\text{x})=-\sum_{\text{x}}\text{p}(\text{x})\text{logp}(\text{x})$$ (9)
  $$\text{S}(\text{x},\text{y})=-\sum_{\text{x},\text{y}}{\text{p}}_{\text{x},\text{y}}(\text{x},\text{y})\text{log}{\text{p}}_{\text{x},\text{y}}(\text{x},\text{y})$$ (10)
  If X and Y were mutually independent, their joint mutual information could be expressed as:
  S(X,Y)=S(X)+S(Y) (11)
2. Kanade Lucas Tomasi (KLT) algorithm: The KLT algorithm was a tracking algorithm based on feature points and belonged to the optical flow method. Target tracking based on the KLT algorithm achieved its purposes of tracking through the matching of feature points; thus, the extraction effects of feature points were related to the accuracy and efficiency of tracking. The KLT algorithm must be performed under the premise of the following three assumptions: (1) constant brightness; (2) continuous-time or small movement displacement; and (3) spatial consistency, similar movements of neighboring points, and keeping adjacent.

Satisfying Hypothesis 1 guaranteed that the target was not affected by brightness. Satisfying Hypothesis 2 guaranteed that the feature points could be corresponding in the target domain. Satisfying Hypothesis 3 guaranteed that all points had the same displacement in the same window. It was defined that the same target appeared in two frames of images I and J. If two points in the image matched, the two points were centered and W was the window with a small gray square difference ∈, and d represented the offset. Generally, the weight function was set as *ω*(*x*) = 1, which was defined as:

$$\in =\iint_{w}{\left[J(x)-I(x-d)\right]}^{2}\omega (x)dx$$ (12)

## 5. Results

### 5.1 The classification results of lumbar vertebra degenerative changes based on Gabor wavelet transformation

The correct segmentation of the intervertebral disc position was the basis for ensuring an effective and accurate algorithm of lumber degeneration classification. In this study, the information of the entire intervertebral discs was extracted by using the elliptical fitting method. The steps of extracting the intervertebral discs were shown in Fig 2. Figure (a) showed the superposition effects of the binary images calculated by the boundary information of the intervertebral discs and the original images. Figure (b) showed the boundary points after the boundary detection of the binary images. Figure (c) showed the effects of elliptical fitting of the obtained boundary points.

**Fig 2:** The information extraction process of intervertebral disc positions. (a) The boundary of intervertebral disc based on Gabor, (b) The detection of boundary points, (c) The elliptical fitting.

In this study, the lumbar degenerative changes in levels 6, 7, and 8 were not found. The classification of the degenerative changes only required two parameters that characterized the grayscale information. In this study, 130 intervertebral discs were successfully fitted, and 109 of them were observed by doctors, including 5 intervertebral disc degeneration in level 2, 70 intervertebral disc degeneration in level 3, 25 intervertebral disc degeneration in level 4, and 9 intervertebral disc degeneration in level 5. Compared with the results of the manual diagnosis, the accuracy of the classification method was 88.3%. In addition, the specificity (SPE), accuracy (ACC), and sensitivity (SEN) of this classification were respectively 89.5%, 92.4%, and 87.6%. The specific classification results were shown in Table 2.

**Table 2:** The classification results of this study.

Evaluating indicator	2	3	4	5	Weighted mean
SPE	100%	85.6%	93.6%	98.0%	89.5%
ACC	98.2%	92.1%	90.2%	95.1%	92.4%
SEN	51.3%	96.3%	81.0%	57.2%	87.6%

### 5.2 The tracking results of the lumbar vertebra body

The mutual information method and KLT algorithm were respectively utilized to track the vertebral body based on the theoretical basis of the vertebral body tracking algorithm. The tracking results of the two methods were respectively shown in Figs 3 and 4. As can be seen from Fig 3, the tracking results of the diagonal points at the 45th frame based on the maximum mutual information method had seriously deviated. Therefore, the above-mentioned maximum mutual information method worked well in the cases of a small number of image sequences, and if the number of image frames was continuously increased, the error would accumulate, and the tracking effects of the images were worse. As can be seen from Fig 4, in the image registration process based on the KLT algorithm, the tracking effects were usually affected by the soft tissue motions. In order to make the accuracy of the registration unaffected, the boundary information of vertebral body was strengthened; after optimization, the soft tissues in the obtained images were smoothened, and the boundary information of the vertebral body was enhanced. The KLT algorithm calculated the transformation relation by fixing the changes of the feature points, and the results were more accurate. Therefore, the tracking effects based on the KLT algorithm were better and faster than those based on the maximum mutual information method.

**Fig 3:** Tracking results of the maximum mutual information method. (a) The 1st frame, (b) The 45th frame.

**Fig 4:** Tracking results of the KLT algorithm. (a) The 1st frame, (b) The 45th frame.

## 6. Discussion

LDH is caused by various factors such as tissue degeneration, long-term strains or injuries, and the rupture of annulus fibrosus in the lumbar intervertebral disc region. The nucleus pulposus of LDH patients would be herniated backward or in a certain direction from the ruptured gap. As the situation is continued, it would result in the stimulation or compression of the nerve root and cauda equina in the corresponding segment and further cause pains in the lower back; some patients may suffer from lower extremity radiation pains. MRI could perform stereoscopic scanning through the horizontal and sagittal positions and could directly observe the vertebral body, the intervertebral discs, the spinal cord, and even the subarachnoid space as well as the adjacent organs and structures. During the diagnosis of LDH, MRI could directly observe the degree of signal changes, determine the locations, directions, and extents of LDH, as well as the relation of nucleus pulposus, nerve roots, and intervertebral discs, and have obvious advantages in the diagnosis of diseases.

The manual analysis of MRI images by doctors is often with subjectivity and low efficiency. Therefore, in this study, the diagnostic values of the feature extraction algorithm in lumbar intervertebral disc degenerative changes were explored through the theoretical basis of Gabor wavelet transformation. First, the Gabor wavelet was introduced, and the information of lumbar intervertebral disc was extracted from MRI images through Gabor wavelet transformation, which could easily and quickly realize the localization of the lumbar intervertebral discs. Through different Gabor coefficients, the annulus fibrosus and nucleus pulposus could be reasonably distinguished, and the accuracy of the results was ensured. The classification method based on Gabor wavelet transformation could effectively classify the lumbar intervertebral disc degenerative changes, and the accuracy rate could reach 88.3%. However, in this study, when comparing with the artificial diagnosis results made by doctors, only the degree of lumbar disc degeneration was compared, and the diagnosis of specific diseases was not analyzed. In subsequent works, LDH could be used as a research disease to achieve the classified detection of diseases by images. Combining the shape of the intervertebral disc with the characteristics of multi-scale and multi-direction of the Gabor filter, the Gabor filter in a specific direction was used to extract the texture features of the intervertebral disc from the MRI image and obtain the information such as the angle, edge, and structure of the intervertebral disc. Supplemented by the prior information of the position relationship between the discs, the positioning of the intervertebral discs was finally realized.

## 7. Conclusions

This study used the Gabor coefficient map to fully utilize the angle information of the intervertebral disc to achieve accurate positioning, indicating that it was a method worth exploring, which could be considered to expand to the entire spine later. In addition, in the classification of degenerative changes in lumbar intervertebral discs, due to the lack of samples, the current algorithm could only be tested in the degenerative samples in the middle region; therefore, samples of different grades could be added in the future to achieve more accurate grading of degeneration in all 8 grades.

## Supporting information

S1 Data (RAR)

S2 Data (RAR)

## References

[1] TetsuhiroI, WatanabeAtsuya, KamodaHiroto, et al Evaluation of Lumbar Intervertebral Disc Degeneration Using T1ρ and T2 Magnetic Resonance Imaging in a Rabbit Disc Injury Model[J]. Asian Spine Journal, 2018, 12(2):317–324. 10.4184/asj.2018.12.2.317 29713414PMC5913024

[2] BatesNM, TianJing, SmiddyWilliam E, et al Relationship between the morphology of the foveal avascular zone, retinal structure, and macular circulation in patients with diabetes mellitus[J]. Scientific Reports, 2018, 8(1):5355 10.1038/s41598-018-23604-y 29599467PMC5876400

[3] HaqIU, NagoakaR, MakinoT, et al 3D Gabor wavelet based vessel filtering of photoacoustic images[J]. Conf Proc IEEE Eng Med Biol Soc, 2016:3883–3886. 10.1109/EMBC.2016.7591576 28269134

[4] OuX, PanWei, ZhangXu, et al Skin Image Retrieval Using Gabor Wavelet Texture Feature[J]. International Journal of Cosmetic Science, 2016, 38(6):607–614. 10.1111/ics.12332 27068932

[5] Soltani BozchalooiI, LiangM. Rebuttal to “On the distribution of the modulus of Gabor wavelet coefficients and the upper bound of the dimensionless smoothness index in the case of additive Gaussian noises: Revisited” by Dong Wang, Qiang Zhou, and Kwok-Leung Tsui[J]. Journal of Sound Vibration, 2018, 420:393–400.

[6] WangC, ShiXiaofeng, LiWendong, et al Oil species identification technique developed by Gabor wavelet analysis and support vector machine based on concentration-synchronous-matrix-fluorescence spectroscopy[J]. Marine Pollution Bulletin, 2016, 104(1–2):322–328. 10.1016/j.marpolbul.2016.01.001 26795119

[7] WangD, ZhouQiang, TsuiKwok-Leung. On the distribution of the modulus of Gabor wavelet coefficients and the upper bound of the dimensionless smoothness index in the case of additive Gaussian noises: Revisited[J]. Journal of Sound & Vibration, 2017, 395(Complete):393–400.

[8] LiangJ, HouZhenjie, ChenChen, et al Supervised bilateral two-dimensional locality preserving projection algorithm based on Gabor wavelet[J]. Signal Image & Video Processing, 2016, 10(8):1–8.

[9] DuranS, CavusogluMehtap, HatipogluHatice Gul, et al Association Between Measures of Vertebral Endplate Morphology and Lumbar Intervertebral Disc Degeneration[J]. Canadian Association of Radiologists Journal, 2017, 68(2):210–216. 10.1016/j.carj.2016.11.002 28216287

[10] KoichiroM, AkedaKoji, TakegamiNorihiko, et al Morphology of intervertebral disc ruptures evaluated by vacuum phenomenon using multi-detector computed tomography: association with lumbar disc degeneration and canal stenosis[J]. Bmc Musculoskeletal Disorders, 2018, 19(1):164-. 10.1186/s12891-018-2086-7 29793459PMC5968599

[11] Torrents-BarrenaJ, PuigD, MelendezJ, et al Computer-aided diagnosis of breast cancer via Gabor wavelet bank and binary-class SVM in mammographic images[J]. Journal of Experimental & Theoretical Artificial Intelligence, 2016, 28(1–2):295–311.

[12] PaholpakP, DedeogullariEmin, LeeChristopher, et al Do modic changes, disc degeneration, translation and angular motion affect facet osteoarthritis of the lumbar spine[J]. European Journal of Radiology, 2018, 98:193–199. 10.1016/j.ejrad.2017.11.023 29279162

[13] GuT, ShiZ, WangC, et al Human bone morphogenetic protein 7 transfected nucleus pulposus cells delay the degeneration of intervertebral disc in dogs[J]. Journal of Orthopaedic Research, 2017, 35(6):1311 10.1002/jor.22995 26218641

[14] XiaoL, NiC, ShiJ, et al Analysis of Correlation Between Vertebral Endplate Change and Lumbar Disc Degeneration[J]. Medical Science Monitor: International Medical Journal of Experimental & Clinical Research, 2017, 23:4932–4938.2903238110.12659/MSM.904315PMC5655151

[15] LiH, YanJia-zhi, ChenYong-jie, et al Non-invasive quantification of age-related changes in the vertebral endplate in rats using in vivo DCE-MRI[J]. Journal of Orthopaedic Surgery & Research, 2017, 12(1):169.2912196010.1186/s13018-017-0669-xPMC5680764

[16] WangJ Q, KaplarZoltan, DengM, et al Thoracolumbar Intervertebral Disc Area Morphometry in Elderly Chinese Men and Women: Radiographic Quantifications at Baseline and Changes at Year-4 Follow-up[J]. Spine, 2017, 43(10):1.10.1097/BRS.000000000000248229112101

[17] EsmaeilS, KamaliFahimeh, SinaeiEhsan, et al Spinal manipulation in the treatment of patients with MRI-confirmed lumbar disc herniation and sacroiliac joint hypomobility: a quasi-experimental study. Chiropractic & Manual Therapies, 2018, 26(1):16.2979625010.1186/s12998-018-0185-zPMC5956754

[18] TschuggA, LenerSara, HartmannSebastian, et al Preoperative sport improves the outcome of lumbar disc surgery: a prospective monocentric cohort study[J]. Neurosurgical Review, 2017, 40(4):597–604. 10.1007/s10143-017-0811-6 28091825PMC5591354

[19] JinhoL, KimJoowon, ShinJoon-Shik, et al Long-Term Course to Lumbar Disc Resorption Patients and Predictive Factors Associated with Disc Resorption[J]. Evidence-Based Complementary and Alternative Medicine, 2017, 2017(133):1–10.10.1155/2017/2147408PMC552346028769985

[20] WangW, HouJ, LvD Y, et al Multimodal quantitative magnetic resonance imaging for lumbar intervertebral disc degeneration[J]. Experimental & Therapeutic Medicine, 2017, 14(3):2078–2084.2896212710.3892/etm.2017.4786PMC5609182

[21] Rodriguez-SotoAna E., BerryDavid B., JaworskiRebecca, et al The effect of training on lumbar spine posture and intervertebral disc degeneration in active-duty Marines[J]. Ergonomics, 2017, 60(8):1–39.2778861910.1080/00140139.2016.1252858

[22] SunZ M, PengmaojiacuoP, XuH H, et al Association of FasL-844T/C gene polymorphism with FasL expression in the nucleus pulposus of degenerative lumbar intervertebral discs[J]. Nan Fang Yi Ke Da Xue Xue Bao, 2017, 37(7):983–987. 2873638010.3969/j.issn.1673-4254.2017.07.23PMC6765517

[23] XiongX, ZhouZ, FiginiM, et al Multi-parameter evaluation of lumbar intervertebral disc degeneration using quantitative magnetic resonance imaging techniques[J]. Am J Transl Res, 2018, 10(2):444–454. 29511438PMC5835809

[24] GriffithJ F, WangY X J, AntonioG E, et al Modified Pfirrmann grading system for lumbar intervertebral disc degeneration[J]. Spine, 2007, 32(24): E708–E712. 10.1097/BRS.0b013e31815a59a0 18007231

